RETRACTED

# RASSF8 downregulation promotes lymphangiogenesis and metastasis in esophageal squamous cell carcinoma

**DOI:** 10.18632/oncotarget.5923

**Published:** 2015-09-30

**Authors:** Lan Zhang, Jian-Hua Wang, Rong-Xin Liang, Shu-Ting Huang, Jing Xu, Lin-Jing Yuan, Long Huang, Yun Zhou, Xing-Juan Yu, Shao-Yun Wu, Rong-Zhen Luo, Jing-Ping Yun, Wei-Hua Jia, Min Zheng

**Affiliations:** ^1^ Department of Gynecology, Guangzhou, P. R. China; ^2^ Department of Pathology, Sun Yat-Sen University Cancer Center; Guangzhou, P. R. China; ^3^ State Key Laboratory of Oncology in South China, Guangzhou, P. R. China; ^4^ Collaborative Innovation Center for Cancer Medicine, Guangzhou, P. R. China; ^5^ Cardiovascular Department, Second People's Hospital of Guangdong Province, Guangzhou, P. R. China; ^6^ Department of Oncology, The Second Affiliated Hospital, Nanchang University, Nanchang, P. R. China

**Keywords:** tumor metastasis, RASSF8, lymphangiogenesis, esophageal cancer

## Abstract

Lymphatic vessels are the major routes of human esophageal squamous cell carcinoma (ESCC) metastasis. Tumor cells secrete pro-lymphangiogenic factors to induce new lymphatic vessels, promoting lymph node metastasis. In this study, we show that RAS association domain family 8 (RASSF8) expression in ESCC clinical samples was inversely correlated with lymph node metastasis and patients survival. Tumor cells with low RASSF8 expression had higher apparent migratory ability, and promoted and lymphangiogenesis both in vitro and in vivo. RASSF8 downregulation enhanced VEGF-C expression and caused subcellular redistribution of p65 in ESCC. Our results show that RASSF8 acts as a tumor suppressor in ESCC and is a potential therapeutic target for preventing lymph node metastasis.

## INTRODUCTION

Human esophageal squamous cell carcinoma (ESCC) is one of the most lethal malignancies worldwide; it ranks fourth among the top 10 cancer-related deaths in China [1, 2]. Despite advances in diagnosis and treatment over past decades, the clinical outcome of ESCC remains poor due to aggressive malignancy and rapid progression. The presence of cancer cells in the lymph nodes is one of the main negative prognostic factors of ESCC [3]. However, the mechanism by which cancer cells reach the lymph nodes remains poorly understood.

Lymphatic vessels are the major routes of tumor metastasis in ESCC. There is accumulating evidence that, despite the preexisting lymphatic vessels, tumor-associated lymphangiogenesis is an important feature of tumor progression and may facilitate cancer cell dissemination to the lymph nodes [4, 5]. Accordingly, numerous clinical studies have demonstrated a significant correlation between lymphatic vessel density and lymph node metastasis. Clinical evidence suggests that the vascular endothelial growth factor (VEGF) family members VEGF-C and VEGF-D are major lymphangiogenic regulators [6]. Higher VEGF-C expression in ESCC is associated with higher peritumoral lymphatic vessel density, increased lymphatic invasion, and increased lymph node metastasis [7, 8]. VEGF-C and VEGF-D stimulate lymphatic vessel sprouting via VEGF receptor (VEGFR)-3 binding, which is expressed in lymphatic endothelial cells to activate downstream extracellular signal–regulated kinase (ERK) and AKT signaling [9]. Inhibiting VEGF-C/VEGFR-3 signaling suppresses tumor lymphangiogenesis and lymphatic metastasis in pre-clinical models and may be a promising strategy for treating ESCC and other cancers [10-13]. Besides lymphangiogenesis, the presence of cancer cells with more motility and invasiveness features also increases the risks of metastasis.

RETRACTED

RASSF8 is one of the four new members in the RAS association domain family (RASSF). Differing from the classic RASSF members (RASSF1–6), which have a C-terminal Sav/RASSF/Hpo (SARAH) domain, RASSF7–10 contain an N-terminal RA domain and lack the SARAH domain [14-16]. RASSF8 is ubiquitously expressed in all major organs and tissues, including the brain, heart, kidney, liver, lung, and other normal adult human tissues. Endogenous RASSF8 is expressed in both the nucleus and the cell membrane, and it promotes cell–cell adhesion by maintaining adherens junction stability [17]. In lung cancer, downregulated RASSF8 increases cell migration and growth, functioning as a tumor suppressor [17, 18]. However, the biological role and clinical significance of RASSF8 in ESCC remain largely unknown.

In this study, we used clinical patient samples and *in vitro* and *in vivo* models to uncover the suppressive role of RASSF8 in ESCC lymphangiogenesis and metastasis. In ESCC, RASSF8 was markedly downregulated at both mRNA and protein level, and correlated with lymph node metastasis, advanced clinical stage, and poor prognosis. RASSF8 knockdown in ESCC cells increased cell invasion ability and promoted lymphatic endothelial cell tube formation and migration; RASSF8 overexpression had the opposite effect. More importantly, downregulated RASSF8 increased VEGF-C expression by promoting the nuclear–cytoplasmic translocation of nuclear factor-κB (NF-κB) p65, leading to lymphangiogenesis and lymphatic metastasis. These results suggest that RASSF8 is a powerful metastatic suppressor and a potential biomarker in the prognostic assessment of ESCC.

## RESULTS

### RASSF8 downregulation correlates with poor prognosis in human ESCC

Western blotting and quantitative real-time PCR revealed lower levels of endogenous RASSF8 in ESCC cell lines as compared with the immortalized esophageal epithelial cell line NE1 (Fig. 1A). *RASSF8* mRNA levels were downregulated in eight ESCC tumor specimens as compared with the paired adjacent non-tumorous tissue (ANT) samples (Fig. 1C). Consistent with this, immunohistochemical staining of 137 ESCC tissues revealed robust RASSF8 expression in the ANT epithelial components; however, RASSF8 expression was significantly downregulated in tumor tissues, particularly those with lymph node metastasis (Fig. 1B). RASSF8 protein levels were inversely correlated with clinical stage (*p* = 0.001; Table 1) and lymph node metastasis (*p* = 0.002; Table 1). Kaplan–Meier survival analysis and log-rank testing showed that patients with lower RASSF8 expression had poor clinical outcomes (*p* = 0.007; Fig. 1D). Univariate and multivariate analyses indicated that low RASSF8 expression was a prognostic factor, but not an independent one, for ESCC outcome (*p* = 0.009; Table 2).

RETRACTED

**Figure 1:** RASSF8 is frequently downregulated in ESCCs **A**., Western blotting (left) and quantitative real-time PCR (right) results showing RASSF8 levels in eight ESCC cell lines and the NE1 immortalized esophageal epithelial cell line. **B**., Representative images of RASSF8 immunochemical staining in ANT and tumor tissues with or without lymph node metastasis (LN+ and LN-, respectively). Bars = 200 μm (left); 50 μm (right). **C**., Quantitative real-time PCR analyses of RASSF8 expression in eight paired primary ESCC tissues and matched ANT tissues. **D**., Kaplan–Meier curves of the overall survival of 137 ESCC patients with high or low RASSF8 expression. The *p*-value was computed by log-rank test. E., RASSF8 protein expression was lower in LN-positive (LN+) specimens than in LN-negative (LN-) specimens (*p* = 0.004). F., Representative staining images of RASSF8 and the lymphatic marker LYVE-1. Arrows indicate LYVE-1–positive lymphatic vessels (left). Correlation of RASSF8 expression and lymphatic vessel density (LVD) was analyzed (right). Bars = 100 μm. IHC, immunohistochemistry.

**Table 1:** Correlation between RASSF8 expression and clinicopathological features in primary ESCC

Variable	RASSF8 expression		*P* value
	Low (%)	High (%)	
Gender			
female	24	17	0.211
male	45	51	
Age, (years)			
<60	39	40	0.785
≥60	30	28	
Differentiation			
1-2	47	48	0.754
3	22	20	
Staging			
I–II a	17	36	0.001*
II b–IV	52	32	
T status			
T1–T2	16	16	0.962
T3–T4	53	52	
Lymph node metastasis			
No	24	42	0.002*
Yes	45	26	
Distant metastasis			
No	60	64	0.243
Yes	9	4	

* *p*-values indicate significance (*p* < 0.05).

**Table 2:** Univariate and multivariate analyses of prognostic variables in patients with ESCC

Variable	Subset	Hazard ratio (95% CI)	*P* value
***Univariate analysis***			
Gender	Male versus female	1.492(0.900-2.473)	0.121
Age, (years)	≥60 versus <60	1.298(0.820-2.054)	0.266
Differentiation	3 versus 1-2	1.316(1.043-1.660)	0.021*
Staging	II b–IV versus I–II a	1.990(1.226-3.233)	0.005*
T status	T3–T4 versus T1–T2	1.874(1.027-3.421)	0.041*
Lymph node metastasis	Yes versus no	1.838(1.163-2.907)	0.009*
Distant metastasis	Yes versus no	2.571(1.266-5.208)	0.009*
Expression of RASSF8	Low versus high	1.887(1.173-3.036)	0.009*
***Multivariate analysis***		
Differentiation	3 versus 1-2	1.407(1.101-1.798)	0.006*
T status	T3–T4 versus T1–T2	2.129(1.129-4.248)	**0.02**

CI, confidence interval.

* *p*-values indicate significance (*p* < 0.05).

RETRACTED

### ESCC lymph node metastasis correlates with downregulated RASSF8 expression at primary site

Immunohistochemical staining of 66 lymph node metastasis–negative and 71 lymph node metastasis–positive tumor tissues demonstrated significantly downregulated RASSF8 in the latter (*p* = 0.004; Fig. 1E). To determine the effect of RASSF8 on lymphangiogenesis, we investigated whether RASSF8 expression in tumors correlated with peritumoral lymphatic vessel density in ESCC. The lymphatic vessels were stained using anti–lymphatic vessel endothelial hyaluronan receptor (LYVE)-1 antibody. As expected, decreased RASSF8 expression in ESCC was significantly correlated with increased peritumoral lymphatic vessel density in ESCC (*p* = 0.002; Fig. 1F). In addition, RASSF8 was downregulated in lymph node metastasis–positive samples as compared with metastasis-negative samples, such as in cervical cancer (NCBI/GEO/GSE26511; *p* = 0.036; Supplementary Fig. 1A) and prostate tumor (NCBI/GEO/GSE6919; Supplementary Fig. 1B). Our results suggest that RASSF8 downregulation may facilitate lymphangiogenesis and lymph node metastasis.

### RASSF8 downregulation enhances ESCC cell motility and invasion *in vitro*

As cell motility and invasion are important factors in cancer metastasis, we constructed RASSF8 overexpression and knockdown cell lines to characterize the effect. Efficiency was detected by quantitative real-time PCR and western blotting (Fig. 2A). RASSF8 downregulation increased ESCC cell migration speed and invasive ability as compared with the control cells (*p* < 0.05). In contrast, RASSF8 upregulation had the opposite effect (*p* < 0.05; Fig. 2B and 2C). These results suggest that RASSF8 downregulation promotes ESCC progression.

**Figure 2:** RASSF8 is essential for ESCC cell motility and invasiveness **A**., Western blotting (top) and quantitative real-time PCR (bottom) analysis of RASSF8 overexpression and RASSF8 knockdown in EC109 and KYSE410 cell lines. **B**., Representative images of wound healing assay showing the motility of RASSF8 overexpression and knockdown cells as compared with the control cells. Bars = 200 μm. **C**., Representative images of Transwell invasion assay showing ESCC cell invasion ability. Bars = 100 μm. *p < 0.05 (Student's *t*-test). NC, negative control.

RETRACTED

### RASSF8 negatively regulates lymphangiogenesis *in vitro* and *in vivo*

As downregulated RASSF8 expression and lymph node metastasis of ESCC are apparently significantly correlated, it suggests that RASSF8 overexpression plays a negative role in lymphangiogenesis. To examine whether RASSF8 downregulation could stimulate tumor lymphangiogenesis, we conducted tube formation and migration assays using human lymphatic endothelial cells (HLECs). HLECs were seeded in the presence of tumor culture supernatants (TSNs) from RASSF8/RASSF8-RNAi (RNA interference)-transfected ESCC cells. RASSF8 inhibited the ability of ESCC cells to induce tube formation and migration, whereas RASSF8 knockdown promoted it (Fig. 3A and 3B).

**Figure 3:** RASSF8 downregulation increases the ability of ESCC cells to induce lymphangiogenesis *in vitro* **A**., Representative images (left) of HLECs cultured on Matrigel-coated plates with TSNs from ESCC cells. Bars = 500 μm. The average number of tube junctions per field was calculated (right). **B**., Representative images (left) and quantification (right) of HLEC migration assay. Bars = 100 μm. Data shown are the mean ± SEM of three fields from three independent experiments. *p < 0.05 (Student's *t*-test). NC, negative control.

We evaluated the effect of RASSF8 on lymphangiogenesis and lymphatic metastasis in ESCC cells using a lymph node metastasis model. EC109 cells stably expressing RASSF8 or RASSF8-RNAi, and control EC109 cells were implanted in the footpads of BALB/c-nu mice. The lymphatic vessel density in the tumors that developed from RASSF8-overexpressing cells was lower than that of tumors from the control cells. Conversely, lymphatic vessel density was significantly increased in tumors formed by RASSF8 knockdown cells (Fig. 4A). In addition, RASSF8 knockdown in the EC109 cells increased popliteal lymph node volume (Fig. 4B) and cytokeratin-positive immunohistochemical staining (Fig. 4C). The ratio of lymph node metastasis was decreased in the EC109-RASSF8 group and increased in the EC109-RASSF8-RNAi group (Fig. 4E).

**Figure 4:** RASSF8 downregulation in ESCC cells promotes lymphangiogenesis and lymph node metastasis **A**., Anti–LYVE-1 antibody immunostaining of lymphatic vessels following ESCC cell inoculation in nude mice footpads. Shown are representative images (left) and quantitative analysis of peritumor lymphatic vessels (right). Bars = 100 μm. **B**., Representative images (left) and volumes (right) of popliteal lymph nodes. **C**., Representative images of anti-cytokeratin antibody−immunostained popliteal lymph nodes from mice inoculated with ESCC cells. Bars = 50 μm. **D**., Ratios of metastatic to total dissected popliteal lymph nodes from mice inoculated with ESCC cells.

RETRACTED

### RASSF8 downregulation increases VEGF-C expression in ESCC

We investigated whether downregulating RASSF8 would increase the expression of VEGF-C, considered the most potent driver of lymphangiogenesis, in ESCC. Immunohistochemical staining of 23 ESCC primary tumors indicated that RASSF8 expression was inversely correlated with VEGF-C expression (*p* = 0.014; R = 0.503; Fig. 5A). Furthermore, protein expression of VEGF-C was downregulated in RASSF8 overexpression ESCC cell culture supernatants, but upregulated in RASSF8 knockdown ESCC cell culture supernatants (Fig. 5B). Accordingly, VEGF-C expression in the mice footpad tumors was significantly increased in RASSF8 knockdown tissues and was decreased in RASSF8 overexpression tissues (Fig. 5C). As VEGF-C induces phosphorylation of the serine kinases AKT and ERK, which promotes HLEC proliferation, migration, and survival [19], we examined the effect of RASSF8-induced VEGF-C expression on AKT and ERK phosphorylation. Phosphorylated (phospho)-AKT (Ser 473) and phospho-ERK (T202/Y204) were dramatically upregulated in HLECs stimulated by TSNs from RASSF8-RNAi–transduced EC109 or KYSE410 cells (Fig. 5D). Importantly, we found that treatment with a PI3K/AKT signaling inhibitor LY294002 or MEK/ERK signaling inhibitor U0126 could reduce the ability of RASSF8 knockdown cells to induce migration and tube formation in HLECs (Fig. 5F and 5G). These results suggest that RASSF8 downregulation increases VEGF-C expression and promotes VEGF-C–induced signaling.

**Figure 5:** RASSF8 downregulates VEGF-C expression in ESCC cells **A**., RASSF8 protein levels are inversely correlated with VEGF-C in clinical ESCC tissues (*n* = 23, *p* = 0.014, R = 0.503). Left: Images of two representative cases. Right: Correlation analyses of RASSF8 and VEGF-C protein expression in 23 human ESCC tissues. Bars = 100 μm. **B**., ELISA of VEGF-C protein levels in the supernatants of the indicated cells. **C**., Immunohistochemical staining detection of VEGF-C protein levels in footpad tumors. Bars = 100 μm. **D**., Western blots of phospho-AKT (p-AKT, Ser 473) and phospho-ERK (p-ERK, T202/Y204) protein levels in TSN-treated human lymphatic endothelial cells (HLECs). **E**., Western blot analysis of phosphor-AKT (Ser374) and phosphor-ERK (T202/Y204) protein expression in HLECs cultured in TSNs derived from RASSF8 knockdown EC109 cells treated with U0126 or LY294002. **F**., **G**., Representative images and quantifications of matrigel tube formation (Bars = 500 μm) and transwell migration (Bars = 100 μm) assays, respectively, of HLECs cultured with TSN from the indicated cell. Error bars indicate the mean±SEM of three independent experiments. *p < 0.05.

RETRACTED

### RASSF8 downregulation enhances NF-κB transcriptional activity and causes subcellular redistribution of p65 in ESCC

We investigated whether RASSF8 is involved in pathway regulation of NF-κB, a critical transcriptional regulator of VEGF-C [20, 21]. We analyzed NF-κB transcriptional activity in RASSF8 overexpression and knockdown ESCC cells with a NF-κB luciferase report plasmid. RASSF8 downregulation significantly increased NF-κB transcriptional activity in both the EC109 and KYSE410 cell lines. By contrast, RASSF8 overexpression attenuated NF-κB transcriptional activity (Fig. 6A). P65 binds to κB sites and transactivates a variety of genes to promote cellular transformation [22]; we examined the effect of RASSF8 on the subcellular distribution of NF-κB p65 in ESCC cells. As expected, nuclear NF-κB p65 expression was significantly decreased in RASSF8 overexpression cells and was increased in RASSF8 knockdown cells (Fig. 6B and 6C), suggesting that RASSF8 downregulation stimulate NF-κB by promoting NF-κB nuclear–cytoplasmic translocation.

**Figure 6:** RASSF8 downregulation causes subcellular redistribution of p65 in ESCC cells **A**., Relative expression of NF-κB luciferase reporter activities in the cells. Data represents percent change in normalized luciferase activity following RASSF8 or RASSF8-RNAi co-transfection relative to the negative control (NC) vector ± SEM from three independent experiments. *p < 0.05. **B**., Western blots of nuclear (nuc), cytoplasmic (cyto), and total NF-κB p65 expression in the cells. Cytoplasmic control, GAPDH; nuclear control, lamin B1. **C**., Quantification analysis of subcellular distribution acquired from western blotting using ImageJ software (Wayne Rashband). Error bars indicate the mean±SEM from three independent exprements. *p < 0.05.

## DISCUSSION

Most epithelial cancers, including ESCC, initiate metastatic growth by disseminating through lymphatic vessels to the draining lymph nodes [4]. Examining metastatic cancer cells in the regional lymph nodes is a main prognostic factor of patient survival and determines the adjuvant therapies selected [3, 23]. Cancer cells can use the lymphatic system to induce a conductive microenvironment for their survival in lymph nodes and at distant metastasis sites [24]. Developing new anti-cancer strategies by targeting the lymphatic system to reduce metastases and improve therapeutic efficiency would be desirable.

RETRACTED

This report presents the first large-scale ESCC clinical study showing a significant clinical association between low RASSF8 expression and poor overall survival. RASSF8 downregulation in cancer cells contributes to increased ESCC cell invasion capacity, as RASSF8 re-expression inhibited cell invasion. Furthermore, loss of RASSF8 in ESCC cells may promote lymphatic endothelium migration and capillary-like tube formation, and *in vivo* tumor lymphangiogenesis and lymphatic metastasis, via VEGF-C upregulation under NF-κB transcriptional control.

VEGF-C and VEGF-D are the most potent regulatory growth factors of lymphatic endothelium proliferation, migration, and survival in human cancers [25, 26]. VEGFR-3 activation induced by VEGF-C or VEGF-D leads to AKT and ERK phosphorylation, which promotes tumor-associated lymphatic vessel growth and enhances lymph node metastasis in many human cancers. Although fibroblast growth factor 2 (FGF-2) [27], insulin-like growth factor 1 (IGF-1) and IGF-2 [28], hepatocyte growth factor (HGF) [29], and platelet-derived growth factor-BB (PDGF-BB) [30] induce lymphangiogenesis in various contexts, most of these effects may be secondary to VEGF-C and VEGF-D induction in inflammatory cells and fibroblasts [31]. VEGF-C upregulation is the main mechanism by which oncogenes or other factors promote lymphangiogenesis and lymphatic metastasis in cancer. Our data suggest that RASSF8 acts on the lymphatic system if VEGF-C increases. The clinical results and *in vitro*/*in vivo* observations demonstrate higher VEGF-C expression and lymphatic vessel density in ESCC tumor tissues with loss of RASSF8. RASSF8 overexpression inhibits VEGF-C expression in ESCC cells, and AKT and ERK phosphorylation in the tumor-associated lymphatic endothelium.

NF-κB, one of the major regulators of VEGF-C, is constitutively activated in ESCC and various cancers [21, 32, 33]. RASSF8 is a negative regulator of NF-κB transcriptional activity in lung cancer [17], where the regulatory protein IκB-α is degraded and p65 dimers enter the nucleus following RASSF8 knockdown in A549 and H1792 cell lines. Our results are consistent with that report: in our study, p65 was upregulated in the nuclei of RASSF8 knockdown ESCC cells and downregulated in RASSF8 overexpression ESCC cells. Luciferase assay suggested that downregulated RASSF8 increases NF-κB activation. The observed NF-κB activation following RASSF8 depletion is the likely cause of the VEGF-C increase in ESCC cells.

RETRACTED

The migration and invasion assays suggested that downregulated RASSF8 might also play a stimulatory role in cell motility, where cell motility was significantly decreased following RASSF8 depletion. RASSF8 colocalizes to the cell–cell adherens junction component β-catenin and binds to E-cadherin [17], a significant epithelial marker in epithelial–mesenchymal transition (EMT). Growing evidence from experimental and clinical studies demonstrate that EMT plays a critical role in tumor invasion and metastasis by endowing cells with a more motile, invasive phenotype [34]. Whether loss of RASSF8 contributes to EMT in ESCC still needs further investigation.

Nevertheless, the molecular mechanisms that lead to RASSF8 downregulation in ESCC have not been fully elucidated. The *RASSF1A* gene is one of the most widely reported epigenetically inactivated genes and could be a useful molecular marker for cancer diagnosis and prognosis [35]. RASSF2, RASSF4, RASSF5, and RASSF6 are also epigenetically inactivated in cancer [14]. However, it is unclear whether epigenetic modifications (i.e., promoter hypermethylation) cause RASSF8 downregulation in ESCC. The European Bioinformatics Institute CpG plot program predicts a 1201-bp CpG island upstream of, and inclusive of, the RASSF8 transcription start site. RASSF8 methylation has been reported in a small subset of leukemia [36]. We speculate that such epigenetic regulation of RASSF8 in ESCC may be possible. The exact mechanism of RASSF8 downregulation in ESCC requires intensive study.

In summary, we used clinical and experimental studies to establish a pro-metastasis role of downregulated RASSF8 in ESCCs. RASSF8 downregulation promoted ESCC metastasis by enhancing cell motility and invasiveness and by increasing lymphangiogenesis via the NF-κB/VEGF-C axis. Our characterization of the functions and mechanism of downregulated RASSF8 will not only increase our understanding of ESCC metastasis, but also presents a new therapeutic target for ESCC treatment.

## MATERIALS AND METHODS

### Ethics statement

This investigation has been conducted in accordance with ethical standards and according to the Declaration of Helsinki and to national and international guidelines, and has been approved by Sun Yat-sen University Medical Ethics Committee.

### Patient information and tissue samples

We enrolled 137 patients diagnosed with ESCC who went esophagectomy and lymphadenectomy at the Sun Yat-sen University Cancer Center from 2002 to 2009. Patients attended follow-up visits regularly; written informed consent was obtained from all patients prior to the study. Two experienced pathologists performed the grading and histopathological subtyping of specimens. Eight fresh ESCC and paired ANT esophageal tissues were collected for quantitative real-time PCR. Table 1 summarizes the clinical information of the samples.

RETRACTED

### RNA isolation and quantitative real-time PCR

Total RNA was isolated from cells and tissues using TRIzol reagent (Life Technologies, Carlsbad, CA, USA) according to the manufacturer's instructions. Reverse transcriptase reactions using MMLV reverse transcriptase reagents (Promega, Madison, WI, USA) were performed according to the manufacturer's protocol. Quantitative real-time PCR was performed using GoTaq qPCR Master Mix (Promega) in a Roche LightCycler 480 II PCR system (Roche Diagnostics, Rotkreuz, Switzerland). Relative gene expression was presented as comparative threshold cycle (2^−ΔΔCt^) values and was representative of at least three independent experiments. Glyceraldehyde-3-phosphate dehydrogenase (GAPDH) and β-actin were used to normalize target gene expression. The reverse transcription–PCR primer sequences are as follows: RASSF8, forward 5′-AAGTATGGGTGGATGGAGTTCAG-3′ and reverse 5′-ATGAGGTGCTAAGTGTCTTTCAG-3′; GAPDH, forward 5′-CTCCTCCTGTTCGACAGTCAGC-3′ and reverse 5′-CCCAATACGACCAAATCCGTT-3′; β-actin, forward 5′-TGGCACCCAGCACAATGAA-3′ and reverse 5′-CTAAGTCATAGTCCGCCTAGAAGCA-3′; VEGF-C, forward 5′-CGGACTCGACCTCTCGG-3′ and reverse 5′-TGGACACAGACCGTAACTGC-3′.

### Immunohistochemistry analysis

Paraffin-embedded, formalin-fixed samples were cut into 4-μm sections. Immunohistochemical staining of ESCC tissue sections was performed using diaminobenzidine (Dako, Copenhagen, Denmark) as the chromogen. Serial sections were labeled with antibodies against RASSF8 (Sigma-Aldrich, St. Louis, MO, USA, HPA038163) and LYVE-1 (Abcam, Cambridge, UK, ab14917), or VEGF-C (R&D System, Inc, Minneapolis, MN55413, USA, AF752). We used an immunohistological reactivity scoring system (H-score) [37, 38] to determine RASSF8 and VEGF-C protein levels in tissue. The H-score takes into account the percentage of positive-staining cells (0–100%) in each staining intensity category (0 to 3+) and computes a final score. The H-score is obtained as follows: (3 × percentage of strong staining) + (2 × percentage of moderate staining) + (percentage of weak staining), yielding an H-score range of 0 to 300. The tissues were divided into high and low RASSF8 expression based on the median value of RASSF8 expression level per slide (Supplementary Fig. 2). The average number of LYVE-1–positive stained lymphatic vessels was counted in two selected vessel hot spots at ×200 magnification. The tissues were divided into high and low lymphatic vessel density based on the average number of LYVE-1-positive stained lymphatic vessels per 0.25 mm^2^.

RETRACTED

### Cell lines

The ESCC cell lines KYSE30, KYSE140, KYSE180, KYSE410, KYSE510, KYSE520 were obtained from Deutsche Sammlung von Mikroorganismen und Zellkulturen (DSMZ), the German Resource Center for Biological Material [39]. EC18, and EC109, and the immortalized esophageal epithelial cell line NE1 were kept in the State Key Laboratory of Oncology in South China, Sun Yat-sen University Cancer Center. The cell lines were cultured in Dulbecco's modified Eagle's medium (DMEM; Life Technologies) supplemented with 10% fetal bovine serum (FBS; Life Technologies) in a 5% CO_2_ atmosphere at 37°C. HLECs were purchased from ScienCell Research Laboratories (Carlsbad, CA, USA) and cultured in endothelial cell medium (ECM; ScienCell Research Laboratories) with 5% FBS and endothelial growth medium supplements (VEGF-C–free).

### Plasmid, transfection, and TSNs

A pcDNA3.1/RASSF8 construct was generated by subcloning the PCR-amplified full-length human *RASSF8* coding sequence into a pcDNA3.1 plasmid. The RASSF8-targeting small interfering RNA (siRNA) sequences are as follows: RNAi#1, forward 5′-CUGGAAGGUACACCCUUAUTT-3′, reverse 5′-AUAAGGGUGUACCUUCCAGTT-3′; RNAi#2, forward, 5′-GGCUCGAAUUCCUGAAAGATT-3′, reverse 5′-UCUUUCAGGAAUUCGAGCCTT-3′. The NF-κB luciferase report plasmid was a gift from Linbai Ye (College of Life Science, Wuhan University, Wuhan, China) [40, 41]. SiRNA or plasmid transfection was conducted using Lipofectamine 2000 (Invitrogen) according to the manufacturer's instruction. At 48 h after transfection, the TSNs were harvested, centrifuged, and stored in aliquots at −80°C. Stable cell lines expressing RASSF8 or RASSF8-RNAi were selected with puromycin for 10 days.

### Western blotting assay

Protein was extracted using a protein extraction kit (KeyGen Biotech, KGP250-2100, Nanjing, China) according to the manufacturer's instructions. The primary antibodies used were anti-RASSF8 (Sigma, HPA038163), anti–VEGF-C (R&D, AF752), anti–phospho-AKT (Cell Signaling, Danvers, MA, USA, 4691S), anti-AKT (Cell Signaling, 4060S), anti–phospho-ERK1/2 (Cell Signaling, 4370P), anti-ERK (Cell Signaling, 9102S), anti-p65 (Cell Signaling, 6956S), anti–β-tubulin (Cell Signaling, 2128S), and anti-GAPDH (Abgent, San Diego, CA, USA). Anti–lamin B1 (KeyGen Biotech, KGAA004-2) was used as the control nuclear protein. Signals were detected using Immobilon Western Chemiluminescent HRP Substrate (Millipore, Billerica, MA, USA) and a Tanon 5200 Luminescent Imaging Workstation (Tanon, Shanghai, China).

### Subcellular fractionation

RASSF8 overexpressing and knockdown cells were subjected to subcellular fractionation using the cytoplasmic and nuclear protein extraction kit (KeyGen Biotech, KGP150), according to the manufacturer's instructions. The efficacy of fractionation was determined via western blotting by stripping the polyvinylidene fluoride membranes and re-probed with LaminB1 as the nuclear control protein and GAPDH antibodies as the cytosolic control. The experiment was performed in triplicate.

RETRACTED

### Wound healing assay

In 95–100% confluent ESCC cultures, we generated wounds with a pipette tip, and obtained images of the wound healing (migration) at the 0h, 24h and 48h.

### Invasion assay

BD Falcon Cell Culture Inserts with 8.0-μm pores (BD Biosciences, Franklin Lakes, NJ, USA) pre-coated with Matrigel (BD Biosciences) were placed in a 24-well plate containing 600 μl 10% FBS/DMEM in the lower chamber. ESCC cells were placed in the upper chamber and incubated at 37°C for 24 h. Cells that migrated to the lower membrane surface were fixed in 1% paraformaldehyde, stained with crystal violet and counted under an optical microscope (× 200 magnification).

### Migration assay

Migration assay was performed using a Transwell chamber (BD Biosciences). HLECs (2 × 10^4^) in serum-free medium were placed in the upper chamber. The lower chambers were filled with the ESCC TSNs. After 10-h incubation, HLECs that passed through the membrane were fixed and stained with crystal violet. The number of cells was counted under a microscope (× 200 magnification) from three randomly chosen fields per membrane, and the average number of cells per field was calculated.

### Tube formation assay

For capillary-like tube formation assays, 75 μl/well Matrigel and 75 μl/well serum-free ECM were mixed and polymerized in a 48-well plate. Then, 2 × 10^4^ HLECs in 100 μl ECM and 400 μl TSNs were incubated on the Matrigel layer in each well. After 4 h, images of the tube formation were obtained using phase-contrast microscopy at ×40 magnification.

### Animal model

BALB/c-nu mice (4–5 weeks old) were purchased from the Guangzhou University of Chinese Medicine Experimental Animal Center (Guangzhou, China). EC109 cells infected with lentivirus RASSF8, RASSF8-RNAi, or vector, negative control were suspended in sterile phosphate-buffered saline with 25% Matrigel and injected into the lower mammary fat pads of the mice (four groups, *n* = 6 per group). After 28 days, the tumors and popliteal lymph nodes were excised and measured. Serial 4.0-μm sections were obtained and analyzed by immunochemical staining with anti–LYVE-1 and anti-cytokeratin antibodies (MXB, Fuzhou, China). The popliteal lymph nodes were estimated using the equation (L × W^2^)/2. The ratios of positive-stained lymph nodes to total lymph nodes were calculated.

RETRACTED

### Enzyme-linked immunosorbent assay

The concentration of VEGF-C was determined by a commercially available VEGF-C ELISA Kit (Cloud-Clone Corp, Houston, TX, USA). Enzyme-linked immunosorbent assay was performed according to the instructions of the manufacturer. Briefly, the cell culture supernatants were added to wells coated with VEGF-C polyclonal antibody, and incubated with biotinylated monoclonal anti-VEGF-C antibody at 37°C for 24 hours. Horseradish peroxidase was used to catalyze the color development, and terminated with stop solution. Absorbance was measured at 450nm. The protein concentrations were determined relative to standard samples.

### Inhibiting signaling assays

The inhibitors of PI3K/AKT signaling LY294002 (Selleck Chemicals, Houston, TX, USA) and of MEK/ERK signaling U0126 (Selleck Chemicals) were dissolved in DMSO respectively at a stock concentration of 10mM and added to cell cultures at a concentration of 10uM. After 24 hours, cell culture supernatants were collected for the HLECs incubation and the transwell migration and matrigel tube formation assays.

### Luciferase reporter assay

Briefly, 2 × 10^4^ ESCC cells were seeded in triplicate in 24-well plates and allowed to settle for 12 h. Cells were transfected with 200 ng NF-κB luciferase reporter plasmid and 10 ng pRL-TK *Renilla* plasmid (Promega) using Lipofectamine 2000. At 24 h after transfection, cells were harvested and luciferase activity was analyzed using a Dual-Luciferase Reporter Assay System (Promega) according to the manufacturer's instructions. Firefly luciferase activity was normalized to that of *Renilla* luciferase as the transfection control.

### Statistical analysis

Statistical analysis was performed using SPSS Standard version 16.0 (SPSS Inc, Chicago, IL, USA). Data are presented as the mean ± standard error of the mean (SEM). Overall survival was defined as the period between the date of surgery to disease-related death. Data were censored at the last follow-up for patients who were disease-free or alive at the time of analysis. Survival functions were examined by Kaplan–Meier analysis. Cox regression analysis was used to assess factors related to survival. Correlation coefficients were computed to measure the degree of association between biomarkers. Data from cell line experiments were assessed by a two-tailed Student's *t*-test. *P*-values < 0.05 were considered significant.

## SUPPLEMENTARY MATERIAL FIGURES


